The article "Effective Remediation Strategy for Xenobiotic Zoxamide by Pure Bacterial Strains, Escherichia coli, Streptococcus pyogenes, and Streptococcus pneumoniae" was retracted in 2024. Reasons: signs of a paper mill; suspected computer-generated content; unreliable results or conclusions; concerns about the data.

# Effective Remediation Strategy for Xenobiotic Zoxamide by Pure Bacterial Strains, *Escherichia coli, Streptococcus pyogenes*, and *Streptococcus pneumoniae*

**DOI:** 10.1155/2020/5352427

**Published:** 2020-11-08

**Authors:** Khuram Shahzad Ahmad, Ayesha Sajid, Mahwash Mahar Gul, Daoud Ali

**Affiliations:** ^1^Department of Environmental Sciences, Fatima Jinnah Women University, The Mall Rawalpindi, Pakistan; ^2^Department of Zoology, College of Science, King Saud University PO Box 2455, Riyadh, 11451, Saudi Arabia

## Abstract

Zoxamide, a class IV hazardous fungicide, is perilous for the environment due to its highly persistent nature. Up till the current date, there are no reports on the biodegradation of zoxamide. The scarcity of knowledge in this domain led to the present research to evaluate the biodegradation of this benzamide fungicide by three bacterial strains, *Escherichia coli* (EC)*, Streptococcus pyogenes* (SPy), and *Streptococcus pneumoniae* (SP). Biotransformation of zoxamide was scrutinized in nutrient broth assemblies for a period of 28 days followed by UV-visible spectrophotometer and GC-MS analysis of the metabolites. The results exhibited a low to medium biodegradation potential of the bacterial cells to metabolize zoxamide. The highest biotransformation percentage was observed by *E. coli* to be 29.8%. The order of half-life calculated for the degradation results was EC (42.5) < SPy (58.7) < SP (67.9) days. GC-MS analysis indicated the formation of several metabolites including, 2-(3,5-dichloro-4-methylphenyl)-4-ethyl-4-methyl-4H-1,3-oxazin-5(6H)-one, 3,5-dichloro-N-(3-hydroxy-1-ethyl-1-methyl--2-oxopropyl)-4-methylbenzamide and 3,5-dichloro-4-methylbenzamide. The research could influence the biotreatment strategies for the environmentally friendly eradication of xenobiotics.

## 1. Introduction

The fungicidal group, benzamide, constrains the development of unwanted wild plants linked with agronomical growth like onion, potato, corn, and ginseng [1]. Zoxamide, (RS)-3,5-dichloro-N-(3-chloro-1-ethyl-1-methyl-2-oxopropyl)-p-toluamide, is applied on weeds and grasses as a preemergent pest control with an administration degree of 5 L/ha [2]. Zoxamide, a relatively recent fungicide, operates by countering the oomycetes [3]. The mode of action of zoxamide is nuclear partition and destruction of the microtubule cytoskeleton [4].

Zoxamide exhibits a low acute toxicity of group IV [5]. Though it is a tenacious skin sensitizer, yet, it is not associated with dermal irritation nor causes any mutation [6] and carcinogenicity in humans [7]. Zoxamide displays mediocre toxicity towards aquatic creatures [8]. Zoxamide dissipation usually occurs through hydrolytic action and photolysis [9]. It is virtually immobilized in terms of its lesser potential for groundwater movement [10]. Research in this field is scarce mainly due to the rigorous, expensive, and inaccessible analytical methods needed to analyze these experiments [11].

The article "Effective Remediation Strategy for Xenobiotic Zoxamide by Pure Bacterial Strains, Escherichia coli, Streptococcus pyogenes, and Streptococcus pneumoniae" was retracted in 2024. Reasons: signs of a paper mill; suspected computer-generated content; unreliable results or conclusions; concerns about the data.

Pesticide mitigation is an imperative issue since the risks concomitant with their usage outweigh the benefits [12]. Unrestrained pesticide usage has ensued in decline of various species including the rare ones [13]. Several environmental compartments have also been effected by their use. Water bodies are affected by pesticides due to their solubility while living species are stimulated through bioamplification [14]. Humans are equally affected by the toxicity of pesticides [15]. It is thus essential to circumvent the hazardous nature of pesticides in effective ways [16].

Biodegradation of zoxamide has not been performed previously. Propyzamide, a benzamide herbicide, has been reported to be degraded by *Comamonas testosteroni* [17]. Assessing the possibility of zoxamide biodegradation by bacterial strains can further contribute to in situ remediation plans. Present research has focused on the use of bacterial strains including, *Escherichia coli, Streptococcus pyogenes*, and *Streptococcus pneumoniae* to elucidate the biotransformation of the fungicide.

## 2. Materials and Methods

### 2.1. Chemicals and Instrumentation

Analytical standard fungicide zoxamide (99% pure), Na_2_SO_4_ (anhydrous), and solvent dichloromethane were utilized. A stock solution of zoxamide (10 mg/L) for the biodegradation experiment was prepared in distilled water. Bacterial culture was prepared in nutrient agar (NA) (Merck, pH 7.0). Pure inoculum of bacterium, *Streptococcus pneumoniae* (SP)*, Streptococcus pyogenes* (SPy), and *Escherichia coli* (EC), were obtained from the Department of Bioinformatics and Biotechnology, International Islamic University, Pakistan. Following instruments were used: weighing balance (AUX220, Shimadzu), incubator (Irmeco, Germany), UV–visible spectrophotometer (BMS-1602), hot plate (MSH-20D, Wisestir instruments), and gas chromatography and mass spectrophotometer (GCMS-QP5050-Schimadzu).

### 2.2. Bacterial Culturing

Pure strains of bacteria, *Streptococcus pneumoniae*, *Streptococcus pyogenes*, and *Escherichia coli* were used as inoculum. Petri dishes, previously sterilized and autoclaved, were utilized for the culturing of strains containing a rich NA medium. Petri plates were sealed with a parafilm tape followed by incubation at 29°C. The entire process of culturing was performed inside a laminar flow hood to protect from contamination. Bacterial colonies were carefully transferred into flasks containing nutrient broth solution for further experimentation [18].

The article "Effective Remediation Strategy for Xenobiotic Zoxamide by Pure Bacterial Strains, Escherichia coli, Streptococcus pyogenes, and Streptococcus pneumoniae" was retracted in 2024. Reasons: signs of a paper mill; suspected computer-generated content; unreliable results or conclusions; concerns about the data.

### 2.3. Zoxamide Biotransformation Assays

Bacterial strains were evaluated for their capability to biodegrade zoxamide in broth assays. Each broth assembly possessed bacterial cells in nutrient broth medium along with zoxamide from the prepared stock solution in 250 mL Erlenmeyer flasks. A control assembly devoid of bacterial cells was also set up. Each assembly was prepared in duplicates. The Erlenmeyer flasks were covered with parafilm tape to avoid entry of other microbes and positioned inside the incubator at 29°C. A constant temperature was provided to the assembly to prevent the effect of temperature variation of the rate of biodegradation. Zoxamide biodegradation was assessed for 28 days. Extractions were performed after every 7 days interval. Pesticide extraction was performed on 7, 14, 21, and 28 days using solvent dichloromethane twice. The extractant was dried using anhydrous sodium sulphate and evaporating to the desired amount. The sample was stored in Eppendorf tubes and stored at −4°C until analysis by UV-spectrophotometer and GC-MS [19].

### 2.4. Biodegradation Analytical Evaluation

Zoxamide degradation in the samples by bacterial cells was evaluated by the following equation (1):

(1) $$\begin{array}{c} S=\left(\frac{\left(a-b\right)}{a}\right)\times 100, \end{array}$$

where *S* is the rate of zoxamide biodegradation in percentage, *a* is the first value of UV-visible absorbance by assembly at *t*_0_, and *b* is the absorbance at various time intervals. *S* has been evaluated in the above equation by the change detected in UV absorbance at various time intervals [20]. The degradation rate was further assessed by applying the first-order reaction kinetics by plotting the graphs of log[*Ct*/*Co*] against number of extraction days. Zoxamide half-life in each assembly was calculated by using equation (2).

(2) $$\begin{array}{c} t_{2}^{1}=0.693/k, \end{array}$$

where *k* is the biodegradation rate constant obtained from the slope of the log plots. Multivariate analysis was performed on the degradation results using Minitab 17 statistical package (US).

The GC-MS evaluation of the samples was performed in a system assembled with a DB-5MS fused quartz capillary column (30 mm × 0.25 mm × 0.25 *μ*m). The source temperature was 180°C, and the transfer line was at 250°C. Injector temperature was maintained at 250°C. The carrier gas was helium at a flow rate of 1.2 mL/min.

## 3. Results

### 3.1. Zoxamide Biodegradation Rate

The biodegradation rate, rate constant, and half-life of zoxamide by bacterial cells are displayed in Table 1. pH was maintained at neutral to avoid the influence of pH change on the rate of biodegradation. Zoxamide biodegradation was evaluated over a span of 28 days. Equation (1) was used to determine the rate of biodegradation by all the bacterial strains. Varying rates of zoxamide reduction were observed by all strains; however, bacterial cells displayed an overall low to medium degradation efficiency over a period of 28 days for zoxamide. First-order reaction kinetics provided degradation rate constants, which were utilized to calculate the half-life by the respective strains. The increasing order of half-life for all the tested bacterial strains is as follows: EC (42.5) < SPy (58.7) < SP (67.9) days. The lowest half-life was observed by *E. coli* strain while the highest was seen by sp. The highest zoxamide biodegradation was observed by EC (29.8%) while the lowest degradation rate was by SP (17.9%). The control sample did not show any significant degradation. First-order reaction kinetics was applied on the degradation rates by all strains. Log plots were produced, and degradation rate constants were obtained from the plots (Figure 1). The biodegradation rate constant was the highest in sample degraded by EC, 0.0163, with the highest degradation percentage, while the lowest rate constant was obtained in sample degraded by SP, 0.0102, with the lowest degradation percentage.

The article "Effective Remediation Strategy for Xenobiotic Zoxamide by Pure Bacterial Strains, Escherichia coli, Streptococcus pyogenes, and Streptococcus pneumoniae" was retracted in 2024. Reasons: signs of a paper mill; suspected computer-generated content; unreliable results or conclusions; concerns about the data.

### 3.2. Metabolite Identification

#### 3.2.1. Escherichia Coli

Degradation results displayed the highest potential of EC to biotransform zoxamide among all the strains. GC-MS analysis was performed for the detection and identification of various metabolites produced as a result of degradation (Figure 2). The transformation products were identified by the NIST library. GC-MS chromatogram displayed the main peak corresponding to the parent compound, zoxamide, at Rt 28.2 min, possessing the highest area percentage, 43%. Another peak corresponding to the bioactive compound, produced by the bacterial cells, was identified at Rt 29.4 min and identified as phenol,2,4-bis(1,1-dimethyl ethyl). The chromatogram also displayed a peak at Rt 27.24 min, which was identified from the NIST library as a transformation compound, 2-(3,5-dichloro-4-methylphenyl)-4-ethyl-4- methyl-4H-1,3-oxazin-5(6H)-one. Peak at Rt 25 min was identified as 3,5-dichloro-N-(3-hydroxy-1-ethyl-1-methyl--2-oxopropyl)-4-methylbenzamide, formed as a result of the ring cleavage of 2-(3,5-dichloro-4-methylphenyl)-4-ethyl-4- methyl-4H-1,3-oxazin-5(6H)-one. The breakage of bond releasing the ethyl and methyl groups from 3,5-dichloro-N-(3-hydroxy-1-ethyl-1-methyl--2-oxopropyl)-4-methylbenzamide resulted in the formation of another metabolite, 3,5-dichloro-4-methylbenzamide, detected at 17.5 min.

The article "Effective Remediation Strategy for Xenobiotic Zoxamide by Pure Bacterial Strains, Escherichia coli, Streptococcus pyogenes, and Streptococcus pneumoniae" was retracted in 2024. Reasons: signs of a paper mill; suspected computer-generated content; unreliable results or conclusions; concerns about the data.

#### 3.2.2. Streptococcus Pyogenes

*Streptococcus pyogenes* was able to exhibit a mediocre degradation of zoxamide. Only 26.7% zoxamide was degraded by SPy. GC-MS chromatogram displayed the peaks corresponding to the parent molecule along with the daughter products produced due to the action of SPy cells on zoxamide. The parent molecule, zoxamide, was detected at Rt 28.2 min. Phenol,2,4- bis(1,1-dimethyl ethyl), a biocompound, was detected at Rt 29 min. The formation of another benzamide ring in the parent molecule resulted in the production of 2-(3,5-dichloro-4-methylphenyl)-4-ethyl-4- methyl-4H-1,3-oxazin-5(6H)-one, which was identified at Rt 27.5 min. Furthermore, the cleaving of the second ring of 2-(3,5-dichloro-4-methylphenyl)-4-ethyl-4- methyl-4H-1,3-oxazin-5(6H)-one resulted in the formation of 3,5-dichloro-N-(3-hydroxy-1-ethyl-1-methyl--2-oxopropyl)-4-methylbenzamide at Rt 26 min.

#### 3.2.3. Streptococcus Pneumoniae

A low degradation rate was observed by the strain *Streptococcus pneumoniae* to be just 17.9%. GC-MS chromatogram displayed a main peak of the parent molecule, while the other peaks were low comparatively. The zoxamide peak was detected at Rt 28.6 min. Phenol,2,4-bis(1,1-dimethyl ethyl), produced by the SP cells, was detected at Rt 30 min. Metabolite, 2-(3,5-dichloro-4-methylphenyl)-4-ethyl-4- methyl-4H-1,3-oxazin-5(6H)-one, was detected at 27.5 min.

### 3.3. Statistical Evaluation

Multivariate analysis was performed on the zoxamide biodegradation results by overlaying the biplot for the degradation percentages of all the bacterial strains (Figure 3). First and second principle components are present in the same plot where the percentages are graphed. The graph displays the point EC to be the farthest from remaining two points indicating the highest degradation percentage, while SP is located closest to the source exhibiting the lowest biodegradation.

## 4. Discussion

Current research explored the potential of three bacterial strains to degrade a fungicide, zoxamide. Among all the strains, only *E.coli* exhibited a mediocre rate of biotransformation of fungicide. The remaining two strains displayed negligible amount of dissipation, which rendered them ineffective to be utilized as bioremedial tools. Although optimal temperature and neutral pH were provided to the strains throughout the experimental duration, yet, SP and SPy failed to provide significant degradation impact on the pesticide.

There are several studies exploring the potential of *E. coli* to degrade aromatic compounds such as phenylacetic acid, 3- and 4-hydroxyphenylacetic acid, phenylpropionic acid, 3-hydroxyphenylpropionic acid, and 3-hydroxycinnamic acid and amines. Due to the superlative potential of *E.coli*, this microbe has been termed as a “model organism” to investigate the metabolism of such compounds. *E. coli* possesses two ring cleavage dioxygenases that catabolise the aromatic structure of pesticide. The ring opening step is a critical step in this scheme. *E. coli* possesses increased solvent tolerance, and hence can degrade the hydrophobic and toxic aromatic compounds. *E. coli* being a facultative microbe can grow in both, presence and absence of oxygen. It is one of the finest microbes at biochemical and genetic level for catabolism of aromatic compounds. Previous studies have displayed that it contains its own set of enzymes and genes for the aromatic molecules' metabolism [21].

The article "Effective Remediation Strategy for Xenobiotic Zoxamide by Pure Bacterial Strains, Escherichia coli, Streptococcus pyogenes, and Streptococcus pneumoniae" was retracted in 2024. Reasons: signs of a paper mill; suspected computer-generated content; unreliable results or conclusions; concerns about the data.

*E. coli* has also been reported to biodegrade pesticides previously. The degradation potential of *E. coli* was seen when it metabolized 70% chlorpyrifos to its transformation product [22]. *E. coli* degrades organophosphorous (pesticides) through the action of phosphonatases [23]. *E. coli* has also displayed the ability to degrade the mixture of pesticides including, DDT, Endrin, and DDE, at about 72% [24]. Chaurasia et al. have displayed the high efficiency of bioengineered *E. coli* to degrade lindane [25].

The bacterial cells utilized in the current experiments have displayed their potential to metabolize zoxamide to some extent. These cells initiate the process of transformation by the cleavage of the carbon and nitrogen bond (Figure 4). This scission results in the formation of an oxidative product. This resulting compound possesses an extra benzene ring in its structure. Further, metabolism by microbes causes the breakage of the ring structure by the bacterial cells. The release of the ethyl and methyl moiety from the molecule further breaks it down into its daughter product with only one ring structure.

## 5. Conclusion

Fungicide zoxamide was analyzed for its biodegradation fate by three bacterial strains, not previously utilized for this purpose. The bacterial cells displayed an overall mediocre transformation rate for the zoxamide metabolism. *Escherichia coli, Streptococcus pyogenes*, and *Streptococcus pneumoniae* degraded zoxamide with half-lives: 42.5, 58.7, and 67.9 days, respectively. Current research scheme can be applicable for the bioremediation of other various hazardous xenobiotics. The present findings are novel and exhibit the utilization of bacterial cells for melioration for the environment.

## Figures and Tables

**Figure 1:** Log plots for the first-order reaction kinetics applied on the biodegradation of zoxamide by bacterial strains.

The article "Effective Remediation Strategy for Xenobiotic Zoxamide by Pure Bacterial Strains, Escherichia coli, Streptococcus pyogenes, and Streptococcus pneumoniae" was retracted in 2024. Reasons: signs of a paper mill; suspected computer-generated content; unreliable results or conclusions; concerns about the data.

**Figure 2:** GCMS chromatograms for zoxamide biodegradation by various bacterial strains (a) *Escherichia coli*, (b) *Streptococcus pyogenes*, and (c) *Streptococcus pneumoniae.*

**Figure 3:** Multivariate biplot for the zoxamide degradation rate by various bacterial strains.

**Figure 4:** Biotransformation pathway initiating from zoxamide ➔ 2-(3,5-dichloro-4-methylphenyl)-4-ethyl-4- methyl-4H-1,3-oxazin-5(6H)-one ➔ 3,5-dichloro-N-(3-hydroxy-1-ethyl-1-methyl--2-oxopropyl)-4-methylbenzamide ➔ 3,5-dichloro-4-methylbenzamide.

**Table 1:** Zoxamide biodegradation percentage, rate constant, and half-life observed by multiple bacterial strains.

Strains	Degradation percentage (%)				Degradation rate constant	Half-life (days)	*R* ^2^
	Day 7	Day 14	Day 21	Day 28			
Escherichia coli	2.15	22.1	26.2	29.8	0.0163	42.5	0.93
Streptococcus pyogenes	4.32	13.5	17.0	26.7	0.0118	58.7	0.89
Streptococcus pneumoniae	3.70	13.6	16.8	17.9	0.0102	67.9	0.73

## Data Availability

No data were used to support this study.
